# All-Cause Death Prediction Method for CHD Based on Graph Convolutional Networks

**DOI:** 10.1155/2022/2389560

**Published:** 2022-07-18

**Authors:** Yutao Xue, Kaizhi Chen, Huizhong Lin, Shangping Zhong

**Affiliations:** ^1^School of Computer and Big Data, Fuzhou University, Fujian 350108, China; ^2^Department of Cardiology, Fujian Medical University Union Hospital, Fujian 350004, China

## Abstract

Coronary heart disease (CHD) has become one of the most serious public health issues due to its high morbidity and mortality rates. Most of the existing coronary heart disease risk prediction models manually extract features based on shallow machine learning methods. It only focuses on the differences between local patient features and ignores the interaction modeling between global patients. Its accuracy is still insufficient for individualized patient management strategies. In this paper, we propose CHD prediction as a graph node classification task for the first time, where nodes can represent individuals in potentially diseased populations and graphs intuitively represent associations between populations. We used an adaptive multi-channel graph convolutional neural network (AM-GCN) model to extract graph embeddings from topology, node features, and their combinations through graph convolution. Then, the adaptive importance weights of the extracted embeddings are learned by using an attention mechanism. For different situations, we model the relationship of the CHD population with the population graph and the K-nearest neighbor graph method. Our experimental evaluation explored the impact of the independent components of the model on the CHD disease prediction performance and compared it to different baselines. The experimental results show that our new model exhibits the best experimental results on the CHD dataset, with a 1.3% improvement in accuracy, a 5.1% improvement in AUC, and a 4.6% improvement in F1-score compared to the nongraph model.

## 1. Introduction

According to the World Health Organization, more than 12 million people die each year as a result of cardiovascular disease. Cardiovascular disease (CVD) is widespread in China. Relevant studies show that the number of people suffering from CVD in China is about 290 million [1], and the mortality rate is higher than that of cancer and other diseases. Coronary heart disease (CHD) is a kind of CVD with a high mortality rate as well as a significant likelihood of recurrence after being cured and discharged from the hospital, all of which are indicators of a bad prognosis.

The pathogenesis of coronary heart disease [2] is due to the continuous accumulation of fat or harmful cholesterol in the arterial wall, which eventually leads to the narrowing and blockage of the arterial wall. The common clinical manifestations of coronary heart disease are arrhythmia, myocardial infarction, and angina pectoris. The mainstream risk factors associated with CHD are a combination of controllable factors (such as lifestyle habits) and uncontrollable factors (such as age, gender, and family history) [3]. The current clinical methods for coronary heart disease detection mainly include [4] ECG, ECG stress test, echocardiography, Holter, hematology, CT angiography, and other technologies. These inspection methods are limited to a certain extent by the personal subjective judgment and long-term experience of doctors.

Establishing an appropriate disease risk assessment model is a critical step in CHD risk assessment and subsequent management decisions. In the past ten years, some medical organizations and institutions have studied disease prediction models based on machine learning (ML) methods [5, 6]. In [7], the authors propose a common collaboration framework (CSHCP). It aims to evaluate people's health through ML technology and provide the best medical plan in a timely manner. Clinically, various physiological indicators of patients with coronary heart disease, such as blood pressure, blood sugar, and cholesterol, will be abnormal. ML methods can accurately uncover hidden factors in the data and perform a prediction of CHD. Giri et al. [8] used the discrete wavelet transform to deconstruct the heart rate signal and four ML classifiers to detect coronary heart disease. Its advantage is that principal component analysis is applied to the wavelet coefficient set to reduce the data dimension. Alickovic et al. [9] extracted features from ECG data using an autoregressive model and used K-nearest neighbors, support vector machines, etc., to distinguish arrhythmia patients from healthy people. Tayefi et al. [10] found that the important variable in CHD is serum hs-CRP level, and they built a prediction model based on a decision tree algorithm. But that limits their expressiveness. D'Ascenzo et al. [11] developed a risk stratification model (PRAISE) for predicting all-cause mortality, myocardial infarction, and postdischarge major bleeding in patients with ACS. However, these previous methods only focus on the differences between clinical features while ignoring the interaction modeling between individual features and global features. Therefore, the high-dimensional nonlinear relationship between the captured features is very limited.

Graph neural networks (GNNs) are a class of methods based on deep learning to deal with the graph domain. It aims to learn low-dimensional vector representations of graphs and nodes by mapping graphs and nodes on graphs to a low-dimensional space by means of artificial neural networks. Scarselli et al. [12] first introduced graph neural networks. However, the disadvantage is that the convolution operation is not considered. Bruna et al. [13] attempted to introduce convolution on graphs and developed spectral graph convolutional networks (GCNs). Defferrard et al. [14] introduced a Chebyshev network (Chebyshev). Kipf et al. [15] simplified the previous method by using only a first-order approximation of the convolution kernel. It enables GCN to directly define convolutions on graphs, providing an end-to-end framework for learning-related tasks.

Recently, graph convolutional neural networks (GCNs) have helped to solve important problems in medicine, especially in the application scenarios of medical images and nonimage information. In some literature, many methodological advances have been made, such as autism and Alzheimer's prediction [16, 17], brain shape analysis [18], pulmonary artery-vein separation [19], mammogram analysis [20], and brain imaging [21]. Graphs provide a powerful and intuitive way to model individuals (nodes) and the relationships or similarities (edges) between individuals. In this scenario, a node can represent the acquired data of a subject at a specific modality or at a specific point in time, and edge weights are used to capture the similarity between each pair of nodes. But there are the following deficiencies: (1) it focuses too much on pairwise similarity between subjects, relying on a single way to construct graphs or edges. (2) GNN may be incapable of learning some deep correlation information between topology and node features. This makes such tasks more challenging and performance limited since they are harder to generalize.

In response to the above challenges, this paper investigates different machine learning techniques to predict the level of uncertainty in CHD based on the risk attributes. In this work, we use a graph neural network approach for the first time to tackle the CHD prediction problem. We used the graph convolution method described by Kipf et al. [15] because of its excellent performance in the node classification task. The main contributions to this paper are as follows:

1. Compared with the past methods of coronary heart disease prediction (naive Bayes, random forest, support vector machine, etc.), we use a new graph convolutional neural network to deal with coronary heart disease.
2. We evaluated two graph construction methods for patients with coronary heart disease, which can automatically construct similarity networks between patients instead of using a single graph structure.
3. A new GCN composite framework is built, which combines the results of different graph channels with the attention mechanism, which is better than the ordinary GCN method.

The rest of this paper is organized as follows: In Section 2, we introduce related methods and models. In Section 3, we will introduce the dataset and conduct experiments. In Section 4, the experimental results are discussed. Finally, Section 5 gives the conclusion.

## 2. Methods

Figure 1 depicts the entire process, from raw data collection to predictive model development and their evaluation process. The risk probabilities of patients with coronary heart disease are determined at the end of the process. The pipeline's three operating steps are data mining and modeling, model construction, and model evaluation.

### 2.1. Graph Convolutional Neural Networks

Graph convolution network (GCN) is a typical GNN model which processes the graph by aggregating the node representation from its neighbors and iteratively updating the representation of each node [15]. Therefore, it is widely used in the supervised and semi-supervised tasks of undirected graphs. Any undirected graph can be expressed as *G*=(*A*,  *X*), where *A* ∈ *R*^*N*×*N*^ is a symmetric adjacency matrix with *n* nodes on a graph, *X* ∈ *R*^*N*×*D*^ is the feature of the input node, and *D* is the dimension of the node feature. If there is an edge between nodes *i* and *j* in the graph, *A*_*i*,*j*_=1; otherwise, *A*_*i*,*j*_=1. The *l*+1 th layer in GCN can be expressed as

(1) $$\begin{array}{c} H^{\left(l+1\right)}=\text{ReLU}\left({\tilde{D}}^{-\left(1/2\right)}\tilde{A}{\tilde{D}}^{-\left(1/2\right)}H^{\left(l\right)}W^{\left(l\right)}\right), \end{array}$$

where *H*^(*l*+1)^ is the output of the *l*+1 th graph convolutional layer, and initially *H*(0)=*X*. Here, $\tilde{A}=A+I$, *A* is the adjacency matrix of the undirected graph, and *I* is the identity matrix. $\tilde{D}$ is the diagonal matrix of $\tilde{A}$. *W*^(*l*)^ is the trainable weight matrix of the *l* th layer, and ReLU is the activation function. When calculating $\hat{A}$, it can usually be simplified to $\hat{A}={\tilde{D}}^{-1/2}\tilde{A}\;{\tilde{D}}^{-1/2}$. For the supervised node classification task, given an arbitrary original graph structure *G*_*ori*_, the embedding of the final output *Z* after a two-layer GCN structure is expressed as

(2) $$\begin{array}{c} Z=f\left(X,A\right)\\ =\text{softmax}\left(\hat{A}\text{ ReLU}\left(\hat{A}{\text{XW}}^{\left(0\right)}\right)W^{\left(1\right)}\right). \end{array}$$

In (2), *W*^(0)^ ∈ *R*^*d*×*nhi*  *d*^ is the weight matrix with a *d*-dimensional feature input to the hidden layer output. *W*^(1)^ ∈ *R*^*nhi*  *d*×*C*^ is a weight matrix from the hidden layer to the *C* class outputs. Define softmax(*x*_*i*_)=exp(*x*_*i*_)/∑_*i*_exp(*x*_*i*_) as the normalizer for all classes. Given input features *X* and topological graph *A*, output labels *Y* are obtained after GCN model training.

### 2.2. Topological Graph Construction Method

#### 2.2.1. Population Graph Construction

The concept of a population graph was first proposed by Parisot in the problem of Alzheimer's disease (AD) and autism spectrum disorder (ASD) disease prediction [22]. Population graphs take advantage of phenotypic information to represent populations as a sparse graph. Define the eigenvectors of the subject of the trainee as its vectorized connectivity matrix. Due to the high dimensionality of the connectivity matrix, a classifier is used to select the most discriminative features from the training set.  Figure 2 illustrates the process of constructing a population graph from CHD data. The population graph *G*=(*V*,  *E*,  *W*) is constructed on the entire population of patients, where |*V*| is *N* nodes, *E* ∈ ℝ^*N*×*N*^ is the edge connection of the graph, and *W* is the weight of the edge. Consider each patient as a node *n*_*i*_ in the graph, consider a set of *H* phenotypic important measures *E*={*M*_*h*_}, and define the adjacency matrix *A*_*p*_ of the population graph as

(3) $$\begin{array}{c} A\left(x_{i},x_{j}\right)=\text{Exp}\left(-\frac{{\left[\rho \left(x_{i},x_{j}\right)\right]}^{2}}{2\sigma^{2}}\right)\cdot \sum_{h=1}^{H}E\left(M_{h}\left(i\right),M_{h}\left(j\right)\right), \end{array}$$

where the Exp function will weight the edges according to the relative distance between the features of each node. If the graph is not fully formed, it will increase the edge weight between the most similar graph nodes. *ρ* is a correlation, which measures the distance between phenotypic measures; *σ* is the mean of the correlation matrix, which determines the width of the kernel. The implication of this similarity measure as in 3 is that patients who belong to the same category (low or high risk) tend to have more similar networks than patients from different categories.

(4) $$\begin{array}{c} E\left(M_{h}\left(i\right),M_{h}\left(j\right)\right)=\left\{\begin{array}{cc} 1, & \text{if }\left|\mu_{i}-\mu_{j}\right|<\beta ,\\ 0, & \text{otherwise.} \end{array}\right. \end{array}$$

In (4), *E*(*M*_*h*_(*i*), *M*_*h*_(*j*)) is the weight matrix, which represents the distance between important measurement indicators, and its size depends on the type of phenotypic important indicator *M*_*h*_ in the graph. *μ*_*i*_ and *μ*_*j*_ are the values of important metrics for nodes *i* and *j*, which are numerically equal to *M*_*h*_(*i*) and *M*_*h*_(*i*). For qualitative indicators such as patient gender, *E* is defined as the delta function *δ*, where *M*_*h*_(*i*)=*M*_*h*_(*j*), *E*(*i*, *j*)=1; otherwise *E*(*i*, *j*)=0. This means that the edge weight between patients with the same phenotypic index is larger. For quantitative indicators such as patient age, *E* needs to be defined as a unit step function about the threshold *β*. And the size of *β* is determined by experience. When *M*_*h*_(*i*) − *M*_*h*_(*j*) is less than the threshold *β*, *E*(*i*, *j*) is increased by 1. In order to maximize the structure of our graphs, we will evaluate the impact of each phenotypic and similarity measure in our experimental section.

#### 2.2.2. KNN Graph Construction

In the field of graph neural networks, the KNN method is often used for data with missing or no graph structure. In this case, we first need to build a K-nearest neighbor graph so that we can apply GCN to extract feature embeddings. We construct the graph according to the idea of K-nearest neighbors (KNNs) [23]. Nodes in the same neighborhood have the most similar features in this graph. The K-nearest neighbor classification is capable of performing discriminant analysis based on uncertainty about the reliable parameters of the probability density. For each sample, we connect the neighbors by finding the top K similar neighbors and setting edges. First, based on the key features of the patient, the similarity between the node features is calculated. The method of calculating the similarity of node features is mainly based on the method of cosine similarity. Specifically, the cosine value between node features *x*_*i*_ and *x*_*j*_ is expressed as

(5) $$\begin{array}{c} \begin{array}{c} S_{i,j}=\frac{X_{i}\cdot X_{j}}{\left|X_{i}\right|\left|X_{j}\right|} \end{array}. \end{array}$$

By calculating the similarity between different vectors, we can get a similarity matrix *S* ∈ *R*^*N*×*N*^ in (5). In this similarity matrix, the cosine similarity between each node *n*_*i*_ and the rest of the nodes *n*_*j*≠*i*_ is recorded. The angle between the vectors is closer to 0° as the cosine value approaches 1, indicating that the two vectors are more similar. Then, select the top *k* most similar node pairs according to the cosine value of each node and set them as edges. In this way, each node has *k* neighbors that are most similar to it. We aggregate this edge information into an undirected K-nearest neighbor graph to get the adjacency matrix *A*_*f*_.

### 2.3. Model

GCN has some weaknesses in fusing node features and topology. To better learn graph embedding information, we refer to and extend the adaptive multi-channel graph convolutional neural network (AM-GCN) [24] architecture. There are three main channels in this model. One is to train the GCN in the original graph channel using the population graph. The other is to use the K-nearest neighbor graph as the input of the feature graph channel to train the GCN. The third is to train the GCN on channels using the common information shared by the original and feature graph. Then, the embeddings trained on the three channels are concatenated, an attention mechanism is used to assign input-specific weight coefficients, and the final embedding is used to predict node classification. The framework of AM-GCN is shown in Figure 3. Algorithm 1 gives the specific process steps.

#### 2.3.1. Multi-Channel Graph Input

In the graph construction method mentioned in Section 2.2, we can get the original topological graph structure through training, which is the population graph and K-nearest neighbor graph, respectively. We take it as the graph branch of the AM-GCN input channel. For the population graph, input the graph (*A*_*p*_, *X*) with the adjacency matrix *A*_*p*_ obtained in the topological space, and the node embedding extracted from the *l*+1 th layer is *Z*_*p*_^(*l*+1)^. For the K-nearest neighbor graph, input the graph (*A*_*f*_, *X*) with the adjacency matrix *A*_*f*_ obtained in the feature space, and the node embedding extracted by the *l*+1 th layer is *Z*_*f*_^(*l*+1)^. Topological space and feature space are not completely unrelated, and the node classification task may be related to the respective information in these two spaces. Therefore, a common channel with parameter sharing is added to the model to share the embedding in the two spaces, and this common embedding is denoted as *Z*_*c*_^(*l*+1)^. The specific calculation method is as follows:

(6) $$\begin{array}{c} Z_{p}^{\left(l+1\right)}=\text{ReLU}\left({\tilde{D}}_{p}^{-\left(1/2\right)}{\tilde{A}}_{p}{\tilde{D}}_{p}^{-\left(1/2\right)}Z_{p}^{\left(l\right)}W_{p}^{\left(l+1\right)}\right), \end{array}$$

(7) $$\begin{array}{c} Z_{f}^{\left(l+1\right)}=\text{ReLU}\left({\tilde{D}}_{f}^{-\left(1/2\right)}{\tilde{A}}_{f}{\tilde{D}}_{f}^{-\left(1/2\right)}Z_{f}^{\left(l\right)}W_{f}^{\left(l+1\right)}\right), \end{array}$$

(8) $$\begin{array}{c} Z_{c}^{\left(l+1\right)}=\frac{\left(Z_{p}^{\prime \left(l+1\right)}+Z_{f}^{\prime \left(l+1\right)}\right)}{2}. \end{array}$$

#### 2.3.2. Attention Mechanism

The channel now has three specifics embedded: *Z*_*p*_, *Z*_*f*__,_ and *Z*_*c*_ (see (6)–(8)). Considering that node labels may be related to one of them or their combination, we use the attention mechanism to learn their corresponding importance (*a*_*p*_, *a*_*f*_, *a*_*c*_), as follows:

(9) $$\begin{array}{c} \left(a_{p},a_{f},a_{c}\right)=\text{Attention}\left(Z_{p},Z_{f},Z_{c}\right), \end{array}$$

where *a*_*p*_, *a*_*f*_, *a*_*c*_ ∈ ℝ^*n*×1^ represents the attention weight of *n* nodes, and the value range of *a* is (0,1). For any node *i*, its embedding in the *i* th row of *Z*_*p*_ is *Z*_*p*_^*i*^ ∈ *R*^1×*h*^. The embedding is transformed by nonlinear transformation, and then a shared attention vector *q* ∈ *R*^*h*′×1^ is used to obtain the attention value *ω*_*p*_^*i*^ as follows:

(10) $$\begin{array}{c} \omega_{p}^{i}=q^{T}\cdot \;\tan\left(W_{p}\cdot {\left(Z_{p}^{i}\right)}^{T}+b_{p}\right). \end{array}$$

In equation (10), *W*_*p*_ ∈ *R*^*h*′×*h*^ is the weight matrix trained by the linear layer, and *b*_*p*_ ∈ *R*^*h*′×1^ is the bias vector of the embedding matrix *Z*_*p*_. Similarly, we can get the attention weight matrix *W*_*f*_,  *W*_*c*_ and attention value *ω*_*f*_^*i*^,  *ω*_*c*_^*i*^ of the embedding matrix *Z*_*f*_,  *Z*_*c*_ for any node *i*. After that, we normalize the attention value *ω*^*i*^ with the softmax function to get the final weights *a*_*p*_^*i*^=softmax(*ω*_*p*_^*i*^), *a*_*f*_^*i*^=softmax(*ω*_*f*_^*i*^)_,_ and *a*_*c*_^*i*^=softmax(*ω*_*c*_^*i*^). Note that the larger the value of *a*, the more important the current embedding is, and the higher the proportion in the final result. For all *n* nodes, there is a learning weight *a*=[*a*^*i*^] ∈ *R*^*n*×1^, and diagonalize the weight as *a*=diag(*a*). Finally, we combine embedding and attention weight to obtain the output *Z*_*a*_ of the attention layer as follows:

(11) $$\begin{array}{c} Z_{a}=a_{p}\cdot Z_{p}+a_{f}\cdot Z_{f}+a_{c}\cdot Z_{c}. \end{array}$$

#### 2.3.3. Objective Function

Here, the output *Z*_*a*_ obtained through the attention layer in (11) is used for a supervised binary classification task with linear transformation and softmax transformation. The task of the model is to predict the classification label $\hat{Y}$, each node *i* has a probability ${\hat{Y}}_{i}$ belonging to the class *C* after transformation, and $\hat{Y}$ can be calculated by way of

(12) $$\begin{array}{c} \hat{Y}=\text{softmax}\left(W\cdot Z_{a}+b\right). \end{array}$$

Assuming that the training set is *L*, the true label corresponding to each piece of data *lϵL* is *Y*_*l*_, and the model predicted label is ${\hat{Y}}_{l}$. For the AM-GCN model, evaluate the cross-entropy error of node classification on all training nodes, denoted by ℒ

(13) $$\begin{array}{c} {ℒ}_{t}=-{\sum_{l\in Y_{L}}\sum_{i=1}^{C}Y_{l}\ln\;\hat{Y}}_{l}. \end{array}$$

Our research on graphs focuses mostly on binary node classification (CHD risk prediction). As a result, we have *C* = 2 in the equation above (Algorithm 1).

#### 2.3.4. Algorithm

The specific algorithm flow is as follows:

*Time Complexity*. It is known that the batch size of model training is *T*, the amount of data is *N*, the number of edges is *ε*, the feature length is *D*, the number of input channels is *M*, the number of output channels is *C*, and the number of hidden layers of the model is *n*, *m*, *k*. The number of two-layer GCN channels is *F*=*n*^2^*m*, and the time complexity of GCN is *O*(*ε*MDF); the time complexity of AM-GCN is *O*(*T*(4*ε*MDF+3*N*^2^*mk*^2^+NMC)) in all training batches.

## 3. Results

### 3.1. Data

The dataset used in this study is real hospital patient data, and the data are partly provided by the Department of Cardiovascular Medicine of a tertiary hospital in Fujian Province, China. In order to protect the privacy and safety of patients, we have removed private data such as the patient's real name, ID number, and mobile phone number.

#### 3.1.1. Dataset

*Description*. The dataset includes data on patients with coronary heart disease collected through follow-up visits during the five-year period from 2016 to 2021. Including 5,850 patients who were discharged from the hospital after surgery, each patient has 430 records of various indicators, and there are about 2,515,500 records in total. But the actual dataset contains a large number of missing patient records, the data are noisy and irregular, and the number of valid records is much lower than this. The dataset consists mainly of structured and unstructured text data. Structured data include basic information such as the patient's age, gender, and living habits. Unstructured text data include patients' ECG examinations, doctors' diagnostic records, and surgical operation records. In general, the content of the dataset can be divided into seven categories: basic patient information, past medical history, electrocardiogram indicators, cardiac color Doppler ultrasound indicators, blood test indicators, medication status, and coronary vascular lesions.  Table 1 shows the clinical and treatment features of the study cohort.  Table 2 shows the patient outcomes of the study data, including healthy and death groups.

The data are expressed as *n* (%), n/*n* (%), or median (IQR). The qualitative index is the proportion of the data, and the quantitative index is the median and the first and third quartiles of the data (25%–75%).

#### 3.1.2. Statistical Analysis

The main predictors varied by study results. Draw a correlation heat map to observe the correlation between multiple features in the data table. The darker the color, the higher the correlation coefficient.  Figure 4 illustrates the associated heat map for the top 14 features.

Figures 5(a) and 5(b), respectively, show the sex distribution histograms of low-risk and high-risk patients with coronary heart disease. Among them, there were 2127 (82.4%) males and 455 (17.6%) females in normal (low-risk) patients after the operation; there were 80 (66.7%) males and 40 (33.3%) females in the death (high-risk) patients.  Figure 5(c) shows a boxplot of the BMI index, where 1 means death (high risk) and 0 means low risk. In the low-risk group, the median BMI was 24.0, the upper quartile (Q3) was 31.3, the lower quartile (Q1) was 17.5, and the number of outliers was 48; in the high-risk group, the median BMI was 24.0, Q3 was 27.3, Q1 was 20.1, and the number of outliers was 10. In the age distribution of patients with coronary heart disease, the median age of the low-risk group is 65, and the number of patients aged 57–71 is the largest, showing a dense distribution; the median age of the high-risk groups is 72, while 63–78 years old is the peak of all-cause death. Figures 5(d) and 5(e) show histograms of patients with coronary heart disease's lifestyle habits (smoking, diabetes history, and hypertension history). 0 means no, 1 means yes, and 0.5 means data loss. The number of smokers in low-risk patients was 1129 (43.9%), and the number of smokers in high-risk patients was 42 (38.5%); the number of diabetics in low-risk patients was 748 (29.4%), while those in high-risk groups were 46 (42.6%); the number of patients with hypertension in low-risk patients was 69 (65.1%), and the number of smokers in high-risk patients was 42 (38.5%).

#### 3.1.3. Data Preprocessing

Data preprocessing ensures the quality of the predicted data by cleaning and transforming the original data so as to obtain high-accuracy results during data analysis and avoid large deviations in the prediction. In the process of Figure 1, we perform the following operations (1–4) on the CHD dataset: (1) is data cleaning. There is a lot of redundant and confusing data in the original phenotype data. We manually screened important factors and eliminated characteristic factors that had little impact on the classification results. We excluded records that were not helpful to the study results, including name, hospital number, and date of surgery, as well as data records of some surgical operations. We initially selected 88 relatively important features. We also included basic variables in this dataset, such as age, gender, BMI, smoking status, diabetes history, and hypertension history, based on relevant research on high-risk factors for coronary heart disease [3]. (2) is data duplication. We select the patient ID number as the unique attribute, delete the data whose ID number does not exist, and keep 5764 valid records. Then, the ID number attribute is deduplicated, a large amount of redundant data is removed, and the patient data record at the latest time point (take the last record as an example) is retained, leaving 4562 pieces of data. (3) is the treatment of missing values and outliers. First, all patients whose information loss rate exceeds 80% are filtered, and the patient data with relatively complete information are retained, with a total of 2702 pieces of data. Then, we process the 88 columns of data features in turn, using the interquartile spacing to detect the abnormal value, setting the default value as the abnormal value, and then setting the upper and lower limits of the standard for the indicators of each feature to restrict the abnormal value. The abnormal value beyond the limit will be replaced by the upper and lower bounds under the current column attribute. (4) is data conversion. The multi-dimensional features of the dataset are discretely distributed, including both qualitative data distribution and quantitative data in different ranges, so the data need to be standardized. We use the Z-score normalization method ($Z=X-\bar{X}/\sigma$) to keep the range of each feature between [0, 1] with a mean of 0 and a variance of 1 to reduce the variance between features.

#### 3.1.4. Risk Factors

The resulting final dataset includes 25 variables: 4 clinical variables (gender, age, BMI, and smoking), 3 medical history variables (diabetes, hypertension, and history of renal insufficiency), 1 electrocardiogram variable (heart rate), 3 cardiac ultrasound variables (E′ wave velocity, left ventricular ejection fraction, and left ventricular weight index), 5 blood test index variables (low-density lipoprotein, total cholesterol, triglyceride, NT-proBNP, and apolipoprotein A), 3 medication status variables (statin, spironolactone, and aspirin), and 6 coronary vascular disease variables (bifurcation site, CTO, angulation, calcification, lesion type, and target vessel).

### 3.2. Experimental Setup

#### 3.2.1. Parameter

The parameters recommended in the study are used to initialize all baseline procedures (see Table 3). Later, we tune their parameters to get the best performance. For each GCN, we train all channels with the same hidden layer size *nhi*  *d*1 and output embedding layer size *nhi*  *d*2, where *nhi*  *d*1 ∈ {16,32,64} and *nhi*  *d*2 ∈ {8,16,32}, respectively. For all neural network models, set the dropout rate to 0.5. Furthermore, for the construction of K-nearest neighbor graphs with different values, we set *k* ∈ {2,…, 9}. We employ the Adam optimizer with a learning rate of 0.001 ~ 0.01 and weight decay ∈{1*e* − 4,5*e* − 4,1*e* − 3,5*e* − 3} throughout training. All experiments are divided into the same intervals on the CHD dataset, that is, 60% training set and 40% test set, and the same random number seed is set in the experimental process to ensure fairness.

#### 3.2.2. Baseline

We compare AM-GCN with other state-of-the-art methods, covering five common non-neural network models in classification and three neural network models. To evaluate the effectiveness of machine learning models on the coronary heart disease dataset, we chose the following representative models as benchmarks for performance comparison, which are implemented through libraries provided by scikit-learn [25], including:

 
*AdaBoost*: The adaptive boosting algorithm (AdaBoost) is an algorithm that iteratively builds strong classifiers [26].
 
*Bayes*: Naive Bayes classifier (NBC) is a widely used classifier algorithm. Here, we choose Bernoulli Bayes [27].
  DT: Decision tree (DT) algorithms use a tree model to identify possible outcomes [28].
  SGD: Stochastic gradient descent (SGD) is a streamlined classifier for fitting linear classifiers under a convex loss function [29].
   SVC: Support vector machines (SVMs) classify data by judging the hyperplanes of the boundary lines between classes in the training data [30].
  DNN: A deep neural network (DNN) is a neural network with multiple hidden layers that update information through backpropagation. Here, we use a multilayer perceptron implementation [31].
  Population-GCN: The graph convolutional neural network (GCN) is a supervised classification model [15] that learns node representations by aggregating adjacent nodes. Here, the graph topology is the population graph, hereinafter referred to as p-GCN.
  KNN-GCN: The graph topology is a K-nearest neighbor graph, hereinafter referred to as K-GCN.
  AM-GCN: The model is introduced in Section 2.3 of this paper.

### 3.3. Performance Metrics

After introducing different machine learning algorithms, we compare the performances of different models for predicting CHD by measuring their performance under different indicators. The evaluation of binary classification models in medicine (cases vs noncases) is based on performance statistics in terms of sensitivity (TP/TP+FN) and specificity (TN/TN+FP), where TP, FP, TN, and FN denote the number of true positives, false positives, true negatives, and false negatives, respectively. We compute and evaluate performance metrics commonly used in classification models [32], such as accuracy, F1-score, AUC (area under the ROC curve), macro-precision, and macro-recall. The receiver operating characteristic curve (ROC) was plotted to understand the relationship between the variables FPR and TPR.

### 3.4. Influence of the Phenotypic(P) Measures

According to the theoretical research in Section 2.2.1, we conduct experiments on different P combinations (sex, age, BMI, smoking) to study the effect of P selection on GCN stability, as shown in Figure 6. The experimental results show that the performance of Acc does not change significantly according to different *P* values, and it fluctuates between 96.4% and 96.7% (±0.3%). In a single-factor study, graphs constructed from the “gender” measure alone achieved decent performance, with an AUC of 85.9% and an F1 of 75.7%. In the two-way combination, the AUC of the measure combination of “gender + age” was 86.8%, and the F1 was 74.7%. The AUC of the measure combination of “gender + BMI” was 86.2%, and the F1 was 75.5%. The AUC of the “age + BMI” combination was 86.0%, and the F1 was 73.7%, which was the worst F1 effect among all combinations. The AUC of the “age + smoking” combination was 87.7%, and the F1 was 75.7%, which was the combination with the best AUC effect. In the multivariate (*H* > 2) measure, the AUC of the combination of “sex + age + BMI” was 86.2%, the F1 was 75.7%, and the effect of the AUC was close to that of the combination of “sex + BMI.” The AUC of the combination of “sex + age + smoking” was 86.9%, and the F1 was 76.1%. The AUC of the combination of “sex + age + smoking + BMI” was 86.4%, and the F1 was 76.1%. From the point of view of AUC and F1, the combination of “age + smoking” in the two-measure factor is the most stable and best overall. For the coronary heart disease population map, we used *H*=2 to maximize the collected information to construct a weighted adjacency matrix (i.e., patient age and smoking similarity) and selected these measures to constitute the population groups for our final prediction task.

### 3.5. Influence of K-Nearest Neighbors

According to the theoretical research in Section 2.2.2, we conduct experiments with different K values (2, ..., 9) to study the influence of the K value on GCN, as shown in Figure 7. The experimental results show that different K values have a slight effect on the performance of Acc, which fluctuates between 96.8% and 97.4% (±0.6%). When K is 2, AUC is 89.4%, F1 is 75.2%, and the effect of F1 is the worst among all possible values of K; when K is 3, AUC is 90.4%, and F1 is 76.2%; when K is 5, AUC is 87.8%, and F1 is 80.9%; when K is 6, AUC is 88.6%, and F1 is 79.0%; when K is 7, AUC is 88.6%, and F1 is 80.0%; when K is 8, AUC is 88.7%, and F1 is 80.4%; when K is 9, AUC is 89.2%, and F1 is 80.0%. Overall, when *K* < 4, the F1 performance dropped significantly compared to the others, which we do not want to see (we want to detect more high-risk patients). As the K value increases, AUC has a slight downward trend, while F1 has a certain room for improvement. At (*K*=9), there is a good AUC and F1, but at the same time, the model training time is also increasing. The value of K represents the number of neighbors of each patient. The larger the value of K is, the number of neighbors allocated to each node increases exponentially (2^*K*^). That is, the composition becomes more complex. For the stability of subsequent experiments, we chose *K* = 6 as the experimental standard for K-nearest neighbor graphs.

### 3.6. Comparison to Other Methods

Experimental results show that AM-GCN has the best performance (see Table 4) in terms of accuracy (97.3%), AUC (90.4%), and F1-score (80.9%). After calculating the F1-score and the area under the ROC curve, it can be observed that AM-GCN performs much better than other machine learning models. A graphical comparison of each model's accuracy, precision, recall, F1-score, and AUC is shown in Figure 8.

## 4. Discussion

The results of the CHD database are shown in Table 4. Among the non-neural network models (AdaBoost, Bayes, DT, SGD, SVC), the accuracy indicator that performs best is the adaptive boosting algorithm, which is 96.0%, and the AM-GCN in this paper is 1.3% higher than it. The best performance of the AUC indicator is the support vector machine, reaching 85.3%, while AM-GCN is 5.1% higher than it. The best F1-score indicator is the adaptive boosting algorithm, reaching 76.3%, and AM-GCN is 4.6% higher than it. The best performer in the recall is the naive SVM, with 75.2%. The best precision performance is the adaptive boosting algorithm, reaching 78.3%, while AM-GCN is 15.1% more effective than it. Among the neural network models (DNN, p-GCN, and K-GCN), the best accuracy indicator is K-GCN, with 97.2% accuracy, while AM-GCN is 0.1% more effective. The best AUC indicator is K-GCN, reaching 88.6%, while AM-GCN is 1.8% better; the best F1-score indicator is K-GCN, reaching 79.0%, while AM-GCN is 1.9% better than it. The best performer in the recall is K-GCN, reaching 71.5%, while AM-GCN is 2.9% better than it. The best performance in precision is K-GCN, reaching 96.5%.

Compared with the nongraph neural network model, the performance of ACC, AUC, and F1 of GCN with appropriate graph structure is better than theirs because GCN has excellent node and edge information aggregation ability, which is not possessed by the nongraph model. In AUC and F1-scores, K-GCN has better performance than p-GCN. The new model combined with p-GCN and K-GCN not only makes up for the shortcomings of two GCNs with different graph structures but also integrates the advantages of the two models. Therefore, the comprehensive performance index is better than the two models without fusion. At the end of our analysis, we present the ROC curve in Figure 9 to visually demonstrate that our proposed algorithm (AM-GCN) shows a higher AUC (90.4%) than other algorithms.

In addition, ROC (receiver operating characteristic) curves were drawn for further study of each machine learning model. The performance of each machine learning model on the research results is visually represented by the ROC in the test set, as shown in Figure 9. The abscissa of the ROC curve is the false-positive rate (or 1-specificity)—the proportion of actual CHD nondeaths identified as deaths by the model, and the ordinate is the true-positive rate (or sensitivity)—the proportion of actual CHD deaths correctly identified by the model. The closer the curve is to the upper left corner, the better the classifier. For a clearer comparison of the differences, we add AM-GCN to the curves. (a) AUCs are predicted by non-neural network models for all-cause mortality. Among them, the AUCs of the adaptive boosting model are 0.80, the AUCs of the naive Bayes are 0.85, the AUCs of the decision tree are 0.75, the AUCs of the stochastic gradient descent are 0.82, and the AUCs of the support vector machine are 0.85. (b) is the AUC predicted by the neural network model for all-cause mortality. Among them, the AUCs of the deep neural network are 0.79, the AUCs of p-GCN are 0.88, and the AUCs of K-GCN are 0.89. In comparison, AM-GCN has an AUC of 0.91, which is the best result.

## 5. Conclusion

In this work, we built a novel neural network model to predict CHD. We employ an attention mechanism to acquire adaptive importance weights for the embeddings while simultaneously extracting unique and common embeddings from topology, node attributes, and their combinations. According to our thorough testing on the dataset, AM-GCN pulls the most essential information from node features and topology and improves classification accuracy by a large margin. Experiments show that the proposed method exhibits better results in various performance metrics compared to several existing baselines. Therefore, the prediction model proposed in this paper is more effective in distinguishing high-risk CHD from low-risk CHD. We found that it can significantly improve the prediction performance, and the excellent prediction ability will optimize its application in the diagnosis and treatment of postoperative recurrence while simplifying the diagnosis process. In the future, we will use more computational techniques to improve the model so that it can predict CHD risk more accurately and effectively.

## Figures and Tables

**Figure 1:** Model development and evaluation pipeline. A flowchart for visualizing the CHD data processing and model development process.

**Figure 2:** Description of the population graph construction process. The basic data are age, gender, BMI, etc.; the indicator data are electrocardiogram, blood drawing and medication records, etc.

**Figure 3:** AM-GCN framework.

**Figure 4:** Correlation heat map.

**Figure 5:** Coronary heart disease patient data analysis. (a), (b) The sex distribution histograms. (c) The BMI index. (d), (e) The histograms of the living habits (smoking, history of diabetes, history of hypertension).

**Figure 6:** The performance of GCN under different combinations of *P* values. (a) Gender; (b) Gender + Age; (c) Gender + BMI; (d) Age + BMI; (e) Gender + Smoking; (f) Age + Smoking; (g) Gender + Age + BMI; (h) Gender + Age + Smoking; (i) Gender + Age + Smoking + BMI.

**Figure 7:** The performance of GCN under different K values. (a) The case of *K* = 2; (b) the case of *K* = 3; (c) the case of *K* = 4; (d) the case of *K* = 5; (e) the case of *K* = 6; (f) the case of *K* = 7; (g) the case of *K* = 8; (h) the case of *K* = 9.

**Figure 8:** Performance comparison of different machine learning models on the CHD dataset.

**Figure 9:** ROC curve for different models of prediction of all-cause mortality. (a) AUC scores for non-neural networks. (b) AUC scores for neural networks.

**Algorithm 1:** AM-GCN-based coronary heart disease risk prediction model.

**Table 1:** Basic information of postoperative patients obtained through follow-up from 2016 to 2021.

Parameters	Before processing (*n* = 5764)	After processing (*n* = 2702)
Age (years)	65 (57–72)	65 (57–72)
Sex (M/F)	4703 (81.6%)	2207 (81.7%)
BMI	24.4 (23.0–25.6)	24.0 (22.7–26.0)
Smoking	1618/5337 (30.3%)	1171/2679 (43.3%)
Diabetes	1600/5301 (30.2%)	794/2650 (30.0%)
Hypertension	2852/5332 (53.5%)	1141/2683 (42.5%)
History of renal insufficiency	63/5309 (1.2%)	26/2673 (1.0%)
Heart rate	69.7 (62.0–76.0)	68 (61.0–76.0)
E ′wave rate	0.06 (0.05–0.14)	0.06 (0.04–0.07)
Left ventricular ejection fraction	59.6 (56.1–66.5)	63.3 (55.1–68.6)
Left ventricular mass index	110.7 (99.0–113.8)	103.4 (86.5–121.0)
Total cholesterol	4.27 (3.43–4.80)	3.95 (3.24–4.85)
Low-density lipoprotein	2.74 (1.98–3.27)	2.48 (1.85–3.28)
Triglycerides	1.57 (1.10–2.54)	1.43 (1.03–2.00)
NT-proBNP	351 (77–866)	129 (37–538)
Apolipoprotein A	1.21 (1.05–1.40)	1.19 (1.04–1.33)
Statins	4104/5265 (77.9%)	2099/2670 (78.6%)
Spironolactone	621/4796 (12.9%)	252/2626 (9.6%)
Aspirin	5113/5194 (98.4%)	2617/2664 (98.2%)

**Table 2:** Patient outcomes.

Result	Category	Before processing (*n* = 5764)	After processing (*n* = 2702)
All-cause mortality	Healthy	5625 (97.6%)	2582 (95.6%)
	Death	139 (2.4%)	120 (4.4)

Before data processing, 139 (2.4%) of 5764 patients died, and 5625 (97.6%) of them were healthy within one year of follow-up; after data processing, 120 (4.4%) of the 2702 records died, and 2582 (95.6%) of the patients were healthy within one year of follow-up.

**Table 3:** Parameter configuration of model.

Parameter name	Parameter value	Parameter description
Epochs	300	Training batch size
lr	0.01	Learning rate
weight_decay	5e-4	Weight decay
K	4	Number of neighbors
nhid1	16	Number of hidden layers 1
nhid2	8	Number of hidden layers 2
Dropout	0.5	Drop rate
Beta	5e-10	Loss function parameter 1
Theta	0.001	Loss function parameter 2
Seed	21	Random number seed
Patience	40	Early stop rounds

**Table 4:** Coronary heart disease dataset prediction results.

Index	Model	Accuracy (%)	AUC (%)	Precision (%)	Recall (%)	F1-score (%)
1	AdaBoost	96.0	79.6	78.3	74.6	76.3
2	Bayes	94.3	84.5	67.2	65.3	66.2
3	DT	95.8	74.7	77.2	73.6	75.2
4	SGD	94.9	82.2	70.9	66.6	68.5
5	SVC	90.1	85.3	61.8	**75.2**	65.3
6	DNN	95.4	78.7	74.2	70.5	72.2
7	p-GCN	96.6	87.7	86.1	70.2	75.7
8	K-GCN	97.2	88.6	**96.5**	71.5	79.0
**9**	**AM-GCN**	**97.3**	**90.4**	93.4	74.4	**80.9**

## Data Availability

The CHD dataset (chd.csv) used to support the findings of this study is restricted by the Institutional Review Board of Fujian Medical University Union Hospital in order to protect patient privacy. Data are available from 569284142@qq.com (HL) for researchers who meet the criteria for access to confidential data.
